RETRACTED

# Assessing the Knowledge and Perceptions of Medical Students After Using Kahoot! in Pharmacology Practical Sessions at King Abdulaziz University, Jeddah

**DOI:** 10.7759/cureus.36796

**Published:** 2023-03-28

**Authors:** Lana Shawwa, Fatemah Kamel

**Affiliations:** 1 Medical Education, King Abdulaziz University, Jeddah, SAU; 2 Pharmacology Department, King Abdulaziz University Faculty of Medicine, Jeddah, SAU

**Keywords:** practical sessions, kahoot, pharmacokinetics, pharmacology, game-based education, active learning

## Abstract

Objective

Game-based e-learning (GbEl) has been shown to motivate students significantly, encourage learning, and improve academic performance. Kahoot! is one such electronic tool, but its implementation and effectiveness in the medical education sector in Saudi Arabia have never been evaluated. In light of this, this study aimed to assess the implementation and efficacy of Kahoot! platform as a learning tool for pharmacology in Saudi Arabian medical education.

Methods

This was a cross-sectional mixed-methods study that employed a quantitative and qualitative approach. It explored the potential of technology-assisted assessment for the interactive learning process using Kahoot! online platform on the participation and performance of 274 Saudi female medical students in their general pharmacology practical sessions during their second year in the Faculty of Medicine (FOM) at King Abdulaziz University (KAU). Data were collected for four one-hour-long pharmacology practical sessions on routes of drug administration, pharmacokinetics (PK) I and II, and drug-drug interactions. The study also explored the perceptions of four faculty members as to how Kahoot! improved students' participation and performance.

Results

Cronbach's alpha value was used to determine the reliability of the questionnaire. Students’ satisfactions with Kahoot! were largely positive. There was a statistically significant difference in the final exam difficulty indexes between topics covered through Kahoot! vs. control sessions. Kahoot! was found to be a practical, agreeable, and interactive formative tool that enhanced student engagement, motivation, and academic achievement. Teachers involved in the study agreed that the advantages of using Kahoot! vastly outweighed the disadvantages.

Conclusion

This study has demonstrated that Kahoot! increased student engagement and motivation, and improved academic achievements in a practical pharmacology course.

## Introduction

Traditionally, pharmacology is taught through lectures in which students are passive recipients of a vast amount of information about drugs and their prescriptions [1]. This didactic approach has been widely used for a long time. Unsurprisingly, medical students largely feel that pharmacology didactic lectures are the most tedious and least valuable of all the learning methods [2].

RETRACTED

Pharmacology is one of the most dynamic and evolving fields in medicine, and it provides a foundation for all physicians in clinical practice. Its scope is vast and broad as a subject, and it encompasses pharmacy as well as experimental and clinical sciences. Medical pharmacology is one of the most fundamental subjects that medical students will have to rely on for the rest of their professional careers. In the second year of medical school, students develop familiarity with patients to understand the clinical aspects of various diseases [1]. Students must learn about numerous drugs, their mechanisms of action, pharmacokinetics, clinical indications, routes of administration, various side effects, contraindications, and many drug interactions. The challenge extends to the faculty teaching pharmacology because there is a need to teach students to make rational therapeutic decisions in clinical scenarios. 

Within the last decade, there has been a huge push for incorporating more active learning strategies in pharmacology education. This prompts the need to explore strategies that create an environment conducive to learning, creative thinking, analysis, and argumentation skills [3]. Lately, gamification has been gaining popularity as an interactive learning strategy that promotes these skills. In 2020, web-based interactive games such as Kahoot! crossword puzzles, instructional videos, music videos, and fill-in-the-blank tables were used as interactive teaching strategies and it was seen that students performed significantly better when fill-in-the-blank activities and videos were utilized [4]. A systematic review has concluded that gamification in healthcare education could improve and help better evaluate the integration of knowledge, comprehension, and confidence in students [5].

In teaching medical content, several studies have demonstrated that game-based e-learning (GbEl) could be an effective tool [6]. 

Kahoot!: gamification for active student learning

Kahoot! is a popular educational game used to develop learners’ skills. It is a free online game that can test students' knowledge. A cell phone, laptop, or Chromebook can be used to run Kahoot! website [7]. Faculty members can create quizzes in a game-based format using multiple-choice questions (MCQs), true-or-false queries, fill-in-the-blanks, etc. The questions can include various multimedia contents, such as pictures or videos, and can be based on real-life scenarios, thereby approximating practice-oriented learning [7].

RETRACTED

A cross-sectional study found that Kahoot! sessions motivated students to study, focus on the essential concepts, and reflect on what they had learned. It was also found to be a promising formative assessment tool in medical education and was recommended for health educators to include in their teaching, particularly for formative assessment [8].

In the Kingdom of Saudi Arabia (KSA), gamification has been successfully used as an educational tool, and many studies have shown its effectiveness in improving student learning [9]. However, most studies have been conducted in school settings and not in college or professional education settings. This study aimed to evaluate the implementation and efficacy of Kahoot! platform as a learning tool for pharmacology in Saudi Arabian medical education. We also intend to add to the existing body of research on the potential of technology-assisted assessment effects of Kahoot! on the perception and academic performance of second-year medical students in their general-pharmacology practical sessions in the Faculty of Medicine (FOM) at King Abdulaziz University (KAU) in Jeddah, KSA. Several questions were addressed in this study: How can Kahoot! be utilized in general-pharmacology practical sessions? How does Kahoot! affect students' academic performance and perceptions? Are students satisfied with the use of Kahoot!? To the best of our knowledge, no previous research has evaluated the effectiveness of Kahoot! in the medical-education sector in KSA, which makes this interventional cross-sectional study the first of its kind.

This article was previously posted to the Research Square preprint platform on October 11, 2021.

## Materials and methods

Kahoot! the game was created by logging into Kahoot! website (http://getkahoot.com). Two instructors in the pharmacology department formulated questions following the sessions' student learning objectives and entered them into the Kahoot! template. One session (on dosage forms) was utilized as a pilot study to validate the quiz. All future sessions would need to be validated because the questions would be different. The first Kahoot! was validated by the instructor and a statistician. An automatically generated code was received. Using their laptops or smartphones, students accessed the game and entered the codes that appeared on the screens to register. Once the Kahoot! started, students earned points based on correct answers and quick responses.

All 274 second-year undergraduate female medical students at FOM, KAU participated. Only female students were included because teaching in FOM, KAU is gender segregated. Data were collected from students in the second semester (from January 2020 until May 2020) for four one-hour-long pharmacology practical sessions on routes of drug administration, pharmacokinetics (PK) I and II, and drug-drug interactions. Practical sessions are part of Pharmacology 201 (PHAM201), spread over 12 weeks in the second semester of the second year of a six-year medical curriculum. It is a basic prerequisite course for the integrated system-based modules taught in the third year of the curriculum. Thus, it provides the students with a foundation in clinical pharmacology. This pharmacology core course aims to train medical students to understand the basic principles of pharmacokinetics and pharmacodynamics, understand the concepts of adverse drug effects and drug-drug interactions, and understand the rational basis of the selection of optimal drugs and dosing regimens based on patient data. The course also includes 10 practical sessions over 18 contact hours.

RETRACTED

The objectives of the practical session that explored routes of drug administration were to identify different routes of drug administration and the advantages and disadvantages of each form. In PK I and II, the students reviewed basic pharmacokinetic parameters, including the volume of distribution, clearance, half-life, steady-state, peak, and trough levels. In the session on drug-drug interaction, students learned about the primary pharmacokinetic mechanisms that underlie drug interactions and the pharmacodynamic characteristics of different drugs, and they identified specific drug-drug interactions that occur commonly in clinical practice.

All practical sessions were taught to all the students in the pharmacology labs, which had an internet connection, and the students had their own electronic devices. The collection of data from 274 female students was based on the principle of ethical conduct. Acting ethically means acting responsibly with integrity and fairness to earn the trust and confidence of all the students to provide a safe environment conducive to learning in a non-discriminatory manner. Test sessions (Kahoot!) involved sessions on routes of drug administration and drug-drug interactions, and the control sessions comprised sessions on PK I and PK II.

A short 10-question pre-test, designed to test knowledge of the session material, was given to all students before each session. They had 10 minutes to answer the questions on their devices. Once the Kahoot! test sessions were over, the quizzes were projected on a large screen to the whole class. The students had to pick what they believed were the correct answers from the displayed list of questions and answers; answering fast and correctly resulted in higher scores. The screen showed a countdown timer and the number of students who answered. After each question, the distribution of students' answers was shown on the screen, showing the level of material comprehension and creating an opportunity to elaborate on questions and answers. After Kahoot! quiz questions were completed, the same 10-question test administered before the session, now referred to as the "post-test," was given to the class to be retaken. At the end of the control sessions, no Kahoot! quizzes were administered, but the “post-tests” were given. Pre- and post-test scores for both Kahoot! and control sessions were collected for analysis.

RETRACTED

Testing in the clinical pharmacology course consisted of two parts. A specific rubric for each practical session was developed for any psychomotor skills, and students were tested on it. The laboratory committee developed this rubric in the pharmacology department. For the theoretical knowledge retained and covered in the practical sessions, an assessment committee in the department created a blueprint and an assessment tool that addressed the course's curriculum learning objectives (CLOs).

In this study, we conducted two types of assessments: assessing retained knowledge and assessing student perceptions toward the use of Kahoot! as an interactive learning strategy. The retained theoretical knowledge was assessed using short answers and matching questions in a summative exam conducted at the end of the practical sessions. This exam was given separately and not included in the final exam because the latter had an MCQ format. Per standard university guidelines, the test’s passing grade was 60%. An 11-item questionnaire was given to the students on the last day of the pharmacology course to assess their perceptions. The questionnaire was intended to establish whether Kahoot! reinforced knowledge and had a positive effect on classroom dynamics. For descriptive statistics, Likert-item responses were used with potential rankings ranging from 5 (strongly agree) to 1 (strongly disagree). 

Additional qualitative data were collected from a faculty focus group comprising four pharmacology faculty members who showed interest in Kahoot!. The principal investigator who conducted the Kahoot! game led the focus group in 20-30-minute discussions on the perceived advantages and disadvantages of Kahoot!. The discussion section summarized the findings of the investigations based on the following aspects: How important is it to play Kahoot! in a classroom? Evaluate the positive sides of Kahoot!. Evaluate the negative sides of Kahoot!. The answers to the three questions were recorded with faculty members’ permission and transcribed by the investigator. After the transcription, a copy was sent to each faculty member to ensure their approval. Thematic analysis to identify the patterns or themes emerging from the faculty focus groups was done based on the Braun and Clarke model (2006) [10].

RETRACTED

Statistical analysis

The quantitative data were entered into the IBM SPSS Statistics version 26.0 (IBM Corp., Armonk, NY). The paired-comparisons t-test was used to compare the mean scores between "pre-" and "post-test" for statistical data analysis, which allowed for the recognition of the magnitude of change in test scores.

The Mann-Whitney U test was used to compare the average participation (summative and final exams) grades between the sessions that utilized the Kahoot! method and those that did not; a p-value <0.05 was considered statistically significant. The questionnaire responses were analyzed with the chi-square test to highlight the association between students' satisfaction with technology-assisted assessment for an interactive learning process using Kahoot! and their final practical exam grades.

## Results

Cronbach's alpha value was used to determine the reliability of the questionnaire, and the validity test was used to evaluate the validity of each item and measure the satisfaction level. As seen in Table 1, the questionnaire was reliable, and all items highly correlated with their intention to measure as evidenced by the validity tests except for item 11.

**Table 1:** Reliability and validity of the questionnaire

Items		Overall scale	Cronbach's alpha
1. Kahoot! was an effective learning tool for me	r	0.836	0.893
2. Kahoot! motivates me to learn more	r	0.832	
3. Kahoot! improved my analytical skills	r	0.755	
4. Kahoot! improved my ability to retain information	r	0.78^*^	
5. I am prepared for tests and quizzes after using Kahoot!	r	0.700	
6. Kahoot! addresses lecture objectives	r	0.760	
7. Kahoot! improved my attendance and participation in lectures	r	0.803	
8. Kahoot! should be utilized in other basic medical sciences	r	0.668	
9. I would like to share this technology with friends and other students	r	0.780	
10. Playing the Kahoot! quizzes was fun. I always looked forward to playing it	r	0.759	
11. The Kahoot! game was a distraction	r	0.244	

Table 2 shows the results of the questionnaire about students’ satisfaction with Kahoot!, which were largely positive.

**Table 2:** Questionnaire about students' satisfaction with Kahoot!

Items	Percentage (%) of students				
	Strongly disagree	Disagree	Not sure	Agree	Strongly agree
Kahoot! was an effective learning tool for me	7.2	5.6	17.4	26.7	43.1
Kahoot! improved my analytical skills	9.2	11.8	23.1	29.2	26.7
Kahoot! improved my ability to retain information	5.1	8.2	16.9	29.2	40.5
Kahoot! improved my attendance and participation in lectures	9.2	9.7	20.0	19.0	42.1
Kahoot! should be utilized in other basic medical sciences	8.7	7.7	17.4	24.1	42.1
Kahoot! addresses lecture objectives	5.6	4.1	21.5	29.7	39.0
Playing Kahoot! quizzes was fun. I always looked forward to playing it	9.2	2.1	14.9	20.5	53.3
I would like to share this technology with friends and other students	8.2	5.1	15.9	24.6	46.2
Kahoot! motivated me to learn more	8.7	7.2	20.0	26.2	37.9
I feel prepared for tests and quizzes after using Kahoot!	20.0	23.6	28.7	13.8	13.8

Table 3 shows the differences in mean improvement scores between Kahoot! and control sessions.

RETRACTED

**Table 3:** Differences in mean improvement scores between Kahoot! and control sessions PK: pharmacokinetics

Parameter	Mean	N	Standard deviation	P-value
Kahoot! drug-drug session improvement	26.56	192	24.37	0.001
Control session: PK 1 improvement	14.19	192	31.49	
Kahoot! drug-drug session improvement	26.23	183	23.85	0.001
Control session: PK 2 improvement	12.39	183	49.59	
Kahoot! route of drug administration improvement	33.89	179	25.04	0.001
Control session: PK 1 improvement	14.53	179	32	
Kahoot! route of drug administration improvement	33.89	179	25.04	0.001
Control session: PK 2 improvement	12.1	179	49.68	

There was a statistically significant difference in the final exam difficulty indexes between topics covered through Kahoot! vs. control sessions as shown in Table 4.

**Table 4:** The differences in the difficulty indexes in the final exam between Kahoot! and traditional classes using student's t-test PK: pharmacokinetics

Parameter		Difficulty index	Mean	P-value
Traditional classes	Pk 1	0.54	0.63	0.0348
	Pk 2	0.71		
Kahoot!	Drug administration	0.99	0.96	
	Drug-drug	0.92		

For the thematic analysis, the six steps explained in Braun and Clarke's (2006) framework were followed:

Step 1: Familiarity with the data: the authors read and re-read the transcript. Initial notes were made: “There is great apprehension on the logistics of applying Kahoot!” and faculty can see the multiple advantages of this game.” Initial ideas about codes emerged. For example: getting feedback on learning, and acceptance by faculty.

Step 2: Generating initial codes: data were organized systematically and meaningfully where similar codes were added together. Following that, each segment of data relevant to the research questions was used for open coding. Coding was done by hand initially. Initial codes that emerged from reading the transcripts were discussed, and preliminary codes were developed. Both researchers coded the transcripts separately, and the codes were later compared. 

RETRACTED

Step 3: Searching for themes: This comprised only four semi-structured interviews conducted by the faculty member using Kahoot!; there was an overlap between the coding stage and identifying preliminary themes. For example, several codes related to effective learning and learners' support were found, and these formed the first theme, i.e., Kahoot! helped the learners share knowledge and support each other through the learning experience. The second theme was that Kahoot! served as a proper tool for formative assessment, as it provided students with an opportunity to learn by getting the wrong answer. Table 5 shows some example responses.

**Table 5:** Example responses

Question	Example response
How important is it to play Kahoot! in a classroom?	“It helps learners share knowledge.” “Learners support each other’s thinking processes.” “Getting the answer wrong is the most effective way of learning through Kahoot!” “The quizzes have emphasized what learners are not good at; they are designed to demonstrate that being wrong is how you learn.”
State the positives of Kahoot!	“If the time given to answering questions was extended, this could help develop high-order thinking.” “They could be a stepping stone to a deeper understanding.” “No fear of answering incorrectly.” “Encourage interest in a new topic.” “Repetition and recall are how Kahoot! can create and consolidate learning.” “The motivation arises from beating scores.” “Detailed report on Kahoot! session easily measures learning impact for each student.”
State the negatives of Kahoot!	“Can’t be applied to cognitive questions (case scenario).” “Internet access (poor signal and technical problems)”

Step 4: Reviewing themes: all data relevant to the themes were gathered. A review of the association of the data with the theme was done.

Step 5: Defining themes: after reviewing and defining the themes, a sub-theme - “student support” - emerged from the formative-assessment-tool theme; after reviewing that, formative assessment might act as a tool to identify students facing academic challenges that need intervention early on from the student-support unit. Examples of thematic codes are presented in Table 6.

**Table 6:** Thematic codes

Themes	Codes
Knowledge support	Share knowledge, support each other’s thinking processes, and develop high-order thinking
Formative assessment tool	Getting the answer wrong and being wrong is how you learn

Step 6: Writing-up: the thematic analysis was reported.

## Discussion

In this study, Kahoot! created a learning experience that was primarily described as “fun” and that contributed to classroom engagement dynamics (in terms of improved participation and motivation to learn). Of note, 64.1% of participants agreed that Kahoot! motivated them to learn more and 61.1% believed that it improved their attendance and participation in class. Several studies have reported that game-based learning is more effective and motivational than traditional ways to promote learning [8]. This difference can be attributed to the interactive nature of game-based learning, which encourages the active involvement of students and stimulates them to learn through active engagement [8]. Moreover, this study endorses research stating that Kahoot! helped students actively engage in their learning activities without it being a distraction [11].

RETRACTED

This study also showed improvement in the scores of students in the “post-tests” versus the “pre-tests” in all Kahoot! sessions compared to control sessions. The detailed student performance reports were made available to the teachers during Kahoot! sessions, allowing them to spot misunderstandings and stimulate feedback and extensive discussions. It also allowed for immediate corrections and facilitated retaining knowledge, as indicated by the final exam results. This distinction of Kahoot! from other formative assessment methods has also been reported by Ismail et al. [12].

Nearly 70% of participants agreed that Kahoot! was an effective learning tool. These results are consistent with the findings of Rondon et al. [6]. It has been reported that Kahoot! helped students focus on relevant content, especially when a large amount of material was taught in lectures. In addition, students have reported that the discussions with teachers during Kahoot! helped them retain information without needing additional revision sessions before tests [13]. Our results are consistent with this report since there was a statistically significant difference in the difficulty indexes in the final exam questions between Kahoot! and traditional sessions. However, an interesting finding in our study was that around 72% of students disagreed or were not sure if using Kahoot! prepared them for tests and quizzes. This finding could be explained by the fact that Kahoot! could only test the recall questions due to the limited number of characters, making it difficult to formulate questions to discern educational learning as per Bloom's taxonomy. However, the questions in our final exam were also recalled ones to match the Kahoot! quiz and the “pre-” and “post-tests.” Another explanation is that students were not aware of the importance of formative assessment as a tool that could help them identify knowledge gaps and better prepare them for exams. This finding has alerted our attention to the need to enlighten students on formative assessments and their role in their exam preparation.

RETRACTED

The advantage of Kahoot!, as perceived by faculty members during the focus-group discussions, was that it promoted the potential for deeper assessment and interactive learning. The faculty also appreciated real-time feedback, which allowed them to measure learning and tailor their instruction based on student understanding of quizzes. The disadvantages were possible problems with internet access and the perception that Kahoot! could not be employed to formulate practice-based scenarios or questions requiring cognitive skills. This could be due to the faculty members’ lack of familiarity with the features of Kahoot!.

Limitations of the study

A significant limitation of this study was that Wi-Fi coverage might have affected internet speed and connectivity and thus impacted students' performance. Also, Kahoot!'s limited number of possible characters for creating questions could have impeded teachers' creativity in formulating more complex questions. In Saudi Arabia, education is gender segregated. Hence, our female principal investigator was only able to use Kahoot! with an all-female cohort of students, limiting the study’s ability to assess the role of gender in terms of motivation and retention of knowledge.

## Conclusions

This study has demonstrated that Kahoot! is a practical, enjoyable, and interactive formative tool that increases student engagement and motivation and improves academic achievements. Therefore, we recommend that medical schools, including KAU, use Kahoot! in lectures, tutorials, and problem-based learning activities for effective formative feedback. Finally, further research on how gaming can foster interpersonal skills, teamwork, professionalism, acceptance of criticism, and verbal and non-verbal communication skills is needed. Also, the use of gaming in non-cognitive skills assessments needs more research.
